# Comparative Efficacy of Robot-Assisted and Laparoscopic Distal Pancreatectomy: A Single-Center Comparative Study

**DOI:** 10.1155/2022/7302222

**Published:** 2022-01-03

**Authors:** Peng Chen, Bin Zhou, Tao Wang, Xiao Hu, Yongqiang Ye, Weidong Guo

**Affiliations:** ^1^Department of Hepatobiliary and Pancreatic Surgery, Heze Municipal Hospital, Heze 274000, Shandong Province, China; ^2^Department of Hepatobiliary and Pancreatic Surgery, The Affiliated Hospital of Qingdao University, Qingdao 266000, Shandong Province, China

## Abstract

**Background:**

Laparoscopic distal pancreatectomy (LDP) has become a routine procedure in pancreatic surgery. Although robotic distal pancreatectomy (RDP) has not been popularized yet, it has shown new advantages in some aspects, and exploring its learning curve is of great significance for guiding clinical practice.

**Methods:**

149 patients who received RDP and LDP in our surgical team were enrolled in this retrospective study. Patients were divided into two groups including LDP group and RDP group. The perioperative outcomes, histopathologic results, long-term postoperative complications, and economic cost were collected and compared between the two groups. The cumulative summation (CUSUM) analysis was used to explore the learning curve of RDP.

**Results:**

The hospital stay, postoperative first exhaust time, and first feeding time in the RDP group were better than those in the LDP group (*P* < 0.05). The rate of spleen preservation in patients with benign and low-grade tumors in the RDP group was significantly higher than that of the LDP group (*P*=0.002), though the cost of operation and hospitalization was significantly higher (*P* < 0.001). The learning curve of RDP in our center declined significantly with completing 32 cases. The average operation time, the hospital stay, and the time of gastrointestinal recovery were shorter after the learning curve node than before.

**Conclusion:**

RDP provides better postoperative recovery and is not difficult to replicate, but the high cost was still a major disadvantage of RDP.

## 1. Introduction

Minimally invasive technology has rapidly developed in recent decades. Laparoscopy has gradually become a routine method in the treatment of kidney, colon, adrenal gland, prostate, and other tumors [1]. Compared with open surgery, laparoscopic surgery has the advantages of fewer complications, less pain, and faster recovery [2]. The pancreas is an important retroperitoneal organ with exocrine and endocrine functions. It locates in a special position where it is adjacent to important organs and large blood vessels while relatively difficult to be exposed and separated during operation [3]. Although minimally invasive pancreatic surgery started later, it has been suggested by the evidence that laparoscopic techniques have been successfully used in patients with inflammatory diseases, trauma, congenital abnormalities, and tumors [4].

Since approximately 50% of pancreatic tumors locate in the body and tail of the pancreas, the main surgical method for such tumors is distal pancreatectomy. According to the tumor types and invasion, lymph node dissection and spleen preservation are selected. Since the first laparoscopic distal pancreatectomy (LDP) was performed more than 20 years ago, it has been recognized as a safe and effective treatment for pancreatic body and tail tumors [5]. Although there is still controversy about the choice of surgical methods for pancreatic malignant tumors, most surgeons still choose minimally invasive surgery for patients with benign and low-grade malignant tumors of the pancreas for they have a longer postoperative survival time. For them, it is important to reduce surgical errors and unnecessary traumas to ensure the quality of life. At the end of the last century, the advent of robotic technology ushered in a new era of minimally invasive surgery. Its high-definition three-dimensional images, more flexible operation angles, and improved ergonomic features do overcome some technical limitations of laparoscopy [6, 7]. However, comparative studies on the efficacy of robotic distal pancreatectomy (RDP) and LDP are rare, especially the follow-up study on the long-term complications caused by partial pancreatectomy and splenectomy.

Despite the rapid promotion and application of robotic surgery in recent years, the high cost of equipment and the professional operation training are still the main obstacles restricting the popularization of this technique [8]. For medical centers with newly introduced robots, even the surgeons with solid laparoscopic technology foundations still need considerable technical trainings and clinical surgery accumulations to master the use of robots proficiently. Moreover, recent reports suggested that robotic surgery may further expand the indications of minimally invasive surgery, which undoubtedly demands surgeons with more professionally clinical and operational experience to complete. The learning curve is the time or the number of operations required for a team or a center to perform surgery proficiently. At present, though literatures about robotic surgical methods boomed, most of which selected the operation time as a single indicator for evaluation, few reports about the learning curve of robotic distal pancreatectomy were provided.

Thus, the objective of this study is to compare the clinical effect and economic cost of RDP and LDP and to investigate the learning curve of RDP procedure primarily.

## 2. Methods

### 2.1. Design and Study Population

This is a retrospective case study. The study was approved by the Hospital Review Committee and followed the guidelines of the Declaration of Helsinki [9]. We reviewed the clinical data of patients who underwent minimally invasive distal pancreatectomy from 2013 to 2019 at the Affiliated Hospital of Qingdao University (Figure 1), including demographic and clinical characteristics, pathological conditions, intraoperative conditions, and short- and long-term postoperative complications. Inclusion criteria: (1) benign, borderline tumors or malignant tumors in the body and tail of the pancreas with clear borders; (2) no severe liver, kidney, heart, and brain dysfunctions; (3) clear imaging data and complete clinical data provided; (4) no macrovascular involvement and distant metastasis; (5) no severe adhesion caused by upper abdominal surgery.

### 2.2. Surgical Technique

Laparoscopic distal pancreatectomy was performed through five ports (one 10 mm port, one 12 mm port, and three 5 mm ports), with the patient in the supine position and a pad under the left side. We used the same trocar positioning for robotic distal pancreatectomy (two 12 mm ports and three 8 mm ports) as described in Figure 2. The surgical procedure is described as follows: After the placement of port and the development of pneumoperitoneum, the gastrocolic ligament was dissected from right to left using the ultrasonic scalpel. If malignant tumors are considered, the distal pancreatectomy and splenectomy should be done. Otherwise, we attempted to preserve the spleen during minimally invasive distal pancreatectomy in patients with benign and borderline pancreatic tumors. Spleen-preserving distal pancreatectomy included transection of the splenic artery and vein, while left gastroepiploic and short gastric vessels were preserved (Warshaw's technique [10]) as well as splenic vessels (Kimura's technique [11]). The preferred technique for splenic salvage was Kimura's technique. If the splenic portal blood vessels are difficult to dissociate, or the spleen blood supply is poor after the severance of splenic portal blood vessels, then the spleen would be excised in combination. We favored parenchymal transection using an endoscopic linear stapler. An ultrasonic device was employed in case of a particularly thick pancreatic gland.

### 2.3. Outcome Evaluation

Diagnostic criteria for pancreatic fistula refer to the definition and classification criteria updated by the International Pancreatic Fistula Research Group in 2016 [12]. Significant clinical pancreatic fistula includes grade B and C fistula. Postoperative hemorrhage of pancreas refers to the definition standard of International Pancreatic Surgery Group [13]. The postoperative complications are classified according to the Clavien–Dindo classification [14], with Clavien–Dindo 3/4 complications counted. The diagnostic criteria of internal and external secretion disorders refer to the definition standard of World Health Organization. Endocrine dysfunction [15]: patients are diagnosed with worsening diabetes, requiring more insulin control or new-onset diabetes. Exocrine dysfunction [16]: fat loss and weight loss (over 3% preoperative weight loss during follow-up), requiring supplementation with trypsin to improve the condition.

### 2.4. Learning Curve Evaluation

The cumulative sum (CUSUM) analysis was employed to evaluate the learning curve of RDP, which is drawn by the MATLAB software. The operation time was selected as the observation indexes. The average of operation was set as the target value. The sequence of operation was taken as abscissa. The cumulative sum of the differences between the operation time and the target value was taken as the ordinate.

### 2.5. Statistical Analysis

All data were analyzed by SPSS 23.0. For continuous variables, the Kolmogorov–Smirnov test was performed first. If normal distribution is satisfied, the independent sample *t*-test is performed for comparison between the two groups. The results are expressed by mean ± standard deviation. Otherwise, the Mann–Whitney U nonparametric test is used for comparison between the two groups, with the results expressed by median (percentile). Classified variables are expressed by frequency (percentage), and the *χ*^2^ test or Fisher exact probability method are used for comparison between the two groups. In the absence of special instructions, *α* = 0.05, that is, the difference was statistically significant when *P* < 0.05.

## 3. Results

A total of 149 patients were enrolled in this study, including 95 cases of LDP and 54 cases of RDP. There was no significant difference in demographic and clinical characteristics between LDP and RDP groups (*P* > 0.05), such as age, sex, BMI, comorbidities, preoperative test indicators, and ASA classification (Table 1). The first postoperative feeding time and flatus time (*P* < 0.05), spleen preservation rate of benign and low-grade malignant tumors (78.3% vs. 50.6%, *P*=0.002), and the splenic arteriovenous preservation rate (50.0% vs. 26.5%, *P*=0.007) of the RDP group were better than those of the LDP group (Table 2). However, the total cost of operation and hospitalization in the RDP group was higher than that in the LDP group (6998.4 ± 1314.9 vs. 3237.7 ± 1442.1, *P* < 0.001; 11522.7 ± 1569.3 vs. 8256.8 ± 2149.0, *P* < 0.001; respectively). No one died during the perioperative period. Serious complications (Clavien–Dindo grade 3/4) and B + C pancreatic fistula accounted for 11 cases (7.4%) and 39 cases (26.2%) in RDP and LDP groups, respectively. There was no significant difference in operation time, intraoperative bleeding volume, and incidence of postoperative complications between the two groups (*P* > 0.05). There were 12 cases (12.6%) of pancreatic ductal adenocarcinoma in the LDP group and 8 cases (14.8%) of pancreatic ductal adenocarcinoma in the RDP group. There was no significant difference in the tumor type, tumor diameter, and R0 resection rate between the two groups (*P* > 0.05) (Table 1).

Twelve of 149 patients were lost to follow-up, and the remaining 137 patients were followed up for 6 to 60 months. Seven patients died of recurrence of tumors, one patient had an overwhelming postsplenectomy infection, 21 patients had postoperative platelet elevation after operation, and no patient had splenic infarction. Among LDP patients, 4 patients with preoperative diabetes mellitus needed to maintain the blood sugar level by increasing insulin injection dosage after operation, and 11 patients had new-onset diabetes mellitus. Two patients suffered from anorexia, dyspepsia, and other pancreatic exocrine disorders, which required long-term use of trypsin preparation to improve the status. Among the patients with RDP, 9 patients had new-onset diabetes mellitus, while no patients had exocrine dysfunction. There was no significant difference in postoperative endocrine and exocrine disorders between the two groups (*P* > 0.05) (Table 3).

The learning curve obtained by cumulative sum analysis is shown in Figure 3, with operative time as the observation index. With the accumulation of surgical cases, the learning curve in Figure 3 exhibited an overall trend of first increasing and then decreasing. The learning curve with operation time as the observation index presented a significant downward trend after 32 cases. To further confirm the above results, 32 cases were selected as the node representing the completion of the learning curve and the clinical data before and after were compared and analyzed. Firstly, the baseline data (age, sex, ASA classification, BMI, preoperative complications, tumor type, tumor diameter, etc.) of the two groups before and after the learning curve node (the first 32 vs. the second 22 cases) were compared, showing no significant difference (*P* > 0.05). After comparing the intraoperative and postoperative indicators of the two groups, it was found that the operation time, hospital stay, and recovery time of gastrointestinal function were shorter after the learning curve node (*P* < 0.05) (Table 4). There was no significant difference between the two groups in pulmonary infection, abdominal infection, incision infection, hemorrhage, pancreatic fistula, spleen-preserving rate, spleen-preserving methods, and the incidence of reoperation (*P* > 0.05) (Tables 4 and 5).

## 4. Discussion

This research of our center showed that RDP had similar indications and safety as LDP. In the present study, 10 patients with LDP underwent conversion, of which 3 cases were due to bleeding, 6 cases were due to difficulty in isolation and exposure, and 1 case was combined with multiple organ resection. On the contrary, none of RDP patients underwent conversion. Studies have reported that patients converted from laparoscopic to open surgery significantly have more severe complications than those not converted [17]. Waters et al. [18] found that the operation time of RDP was longer than that of LDP. The average operation time of RDP in our center was 244 minutes, and there was no significant difference compared with LDP of 227 minutes. However, the average operation time of RDP after the learning curve node decreased from 262 minutes to 217 minutes, which was closer to that of LDP. Although RDP has some disadvantages such as loss of tactile feedback, complex surgical preparation, and other factors that prolong the operation time, its higher spleen preservation rate, more flexible operation, and energy saving for surgeons undoubtedly offset these disadvantages. With the improvement of surgical proficiency, operation time is no longer a limiting factor for the development of RDP, which is also confirmed by the latest systematic retrospective analysis [19]. Compared with patients in the LDP group, the patients in the RDP group have a faster recovery of gastrointestinal function and a shorter hospital stay. There was no significant difference between LDP and RDP patients in the incidence of postoperative complications, including infection, bleeding, pancreatic fistula, and severe postoperative complications such as Clavien–Dindo grade 3–4 complications. Thus, it indicates that RDP still has certain advantages. In terms of total hospitalization cost, especially the surgical cost, RDP does bring certain economic pressure to patients. It is consistent with the results of Kang et al. [20, 21]. According to current research, shortening hospital stay and operation time does not bring significant cost reduction.

The spleen is the most common organ removed in distal pancreatectomy, of which the removal is often optional or unexpected. Successful spleen preservation is one of the keys to minimally invasive distal pancreatectomy, which ensures normal function of the immune system [22]. Patients after splenectomy are more prone to complications such as overwhelming postsplenectomy infection (OPSI), thrombosis, platelet elevation, and increased cancer risk, all of which are inconducive to postoperative recovery and long-term prognosis [23]. For benign, borderline and low-grade malignant noninvasive tumors in the body and/or tail of the pancreas, distal pancreatectomy with spleen preservation should be preferred [24]. However, the preservation of spleen for malignant tumors in the pancreatic body and/or tail remains controversial [25]. At present, there are two internationally recognized methods of spleen preservation, i.e., Warshaw's technique and Kimura's technique. Studies have shown that Kimura's technique is more conducive to the postoperative recovery of patients and the reduced incidence of related complications [26]. Goh et al. [27] found that the spleen-preserving rate of distal pancreatectomy in the robotic group was superior to that of the laparoscopic group, which was contrary to the results of Butturini et al. [28]. Our study suggested that the spleen-preserving rate of the RDP group reached 78.3%, significantly higher than that of the LDP group (50.6%). Moreover, the rate of spleen preservation was especially higher in the RDP group using Kimura's technique. The reasons for the higher spleen preservation rate in the RDP group are probably the clear 3D vision, the more flexible manipulator arm, and the elimination of hand tremor, all of which facilitate the separation of small arterial and venous branches from splenic arteries and veins [29]. Nevertheless, large-scale, prospective randomized controlled trials are needed for the further investigation on the controversy about the spleen preservation rate. The results of our study suggest that effective spleen preservation and/or spleen vessels preservation are indeed important advantages of robotic surgery if surgery and hospital cost are not a major concern for patients.

Robotic pancreatic surgery started relatively late. The CUSUM analysis adopted in this study is a relatively mature method to explore the learning curve of surgery. It calculates the cumulative sum of the differences between the observed value and the target value of the observation indexes in the process of skill acquisition and can accurately judge the variation of the learning curve. In this study, the learning curve was established based on operation time, which stabilized gradually and showed a significant downward trend after 32 cases. By comparing the clinical data of patients, it was found that the operation time and hospital stay of patients became shorter after crossing the learning curve node. The whole learning curve shows several twists and turns, while the plateau is not prominent. It can be inferred that the three stages of the learning curve may not appear regularly. It is because that several factors may influence the analysis, such as (1) the existing differences between individual patients such as pathological type, tumor size, and tumor specific location, despite that there is no difference in the overall baseline data of patients; (2) the cooperation between the master surgeon and the assistant; and (3) exchange of surgical assistants. By searching the literatures about RPD at home and abroad, three studies [30–32] involving the learning curve were found, which showed different nodes in the learning curve. In addition to the study of Benizri et al. using comprehensive factors to analyze the learning curve, the other two studies all analyzed the curve only based on the variable of operation time. The learning curve nodes in Benizri's and Napoli's studies were 7 and 10, respectively, while Zureikat's study showed similar results to our center. Further analysis revealed that there were significantly more bleeding volume, conversion rate, and complication incidence in Benizri's studies than in other studies, probably resulting from their earlier time of operation and lack of multicenter experience. On the contrary, the medical center of Napoli's study had nearly ten years of robotic operation experience, while the medical centers of Zureikat's study and ours all had rich experience in laparoscopic operation before RDP. It indicates that the accumulation of surgical experience or the popularization of surgical methods will affect the time of the appearance of the learning curve node. Thus, it is necessary to comprehensively evaluate the learning curve in combination with various factors of surgery.

Our study still has some limitations. First, there is inherent bias in retrospective cohort studies. Despite many methods such as propensity matching (PSM), the baseline level of the study subjects is still not as effective as that of the randomized controlled trials. Furthermore, the limited single-center data lead to the extreme values of operative time, bleeding volume, postoperative complications, etc. Finally, the comparison of the two surgical procedures lacked empirical consistency. Therefore, high-quality randomized controlled trials would be more convincing for a more comprehensive and systematic comparison between RDP and LDP. Up to now, no randomized controlled trials has been reported for minimally invasive pancreatic surgery. Only a few single-center or multicenter cases were analyzed retrospectively and reviewed systematically [33].

In conclusion, RDP and LDP have similar indications and safety. In general, RDP is not inferior to LDP. Specifically, there was no significant difference in the long-term prognosis of endocrine and exocrine functions between the two groups. Compared with the LDP group, the patients of the RDP group showed a higher success rate, faster recovery rate, and higher rate of spleen preservation for benign and borderline tumors, suggesting a better prognostic effect and quality of life. However, the higher cost is still the main problem need to be solved in robotic surgery. The learning curve of robotic surgery reflects the learning process of a surgical team mastering the technique. Analyzing the learning curve comprehensively is not only helpful to further improve the prognosis of patients but also beneficial to provide reference for other medical centers.

## Figures and Tables

**Figure 1:** Flow chart showing patient enrolment and surgical treatment strategies.

**Figure 2:** Port placement for RDP (a) and LDP (b). C, camera port; R1–R3, robot arm ports; A1, assistant ports.

**Figure 3:** The CUSUM curve according to the operation time. The decreasing point for the operation time begins at the 32nd operation.

**Table 1:** Baseline characteristics, pathology data, and outcomes of patients (MIPD).

	LDP (*n* = 95）	RDP (*n* = 54）	*P*
Age, years, (mean ± SD)	51.74 ± 15.90	50.06 ± 14.77	0.525
Sex, *n* (%)			
Male	29 (30.5)	16 (29.6)	
Female	66 (69.5)	38 (70.4)	0.909
BMI, kg/m^2^, (mean ± SD)	24.23 ± 4.60	24.23 ± 3.59	0.995
CA199, u/ml, median (IQR)	11.0 (7.4–24.5)	12.1 (8.3–17.2)	0.941
CEA, ng/ml, median (IQR)	1.4 (1.0–2.3)	1.4 (0.7–2.3)	0.430
CA125, u/ml, median (IQR)	12.6 (8.2–17.2)	13.6 (11.3–19.6)	0.118
Albumin, g/l, median (IQR)	41.9 (40.0–44.9)	42.2 (40.8–44.4)	0.605
HB, g/l, median (IQR)	132.0 (125.5–146.0)	129.5 (120.0–137.0)	0.119
PDD, *n* (%)	2 (2.1)	4 (7.4)	0.190
Comorbidities, *n* (%)			
Hypertension	22 (23.2)	11 (20.4)	0.694
Diabetes	15 (15.8)	4 (7.4)	0.140
ASA, *n* (%)			
ASA 1	15 (15.8)	7 (13.0)	
ASA 2	52 (54.7)	39 (72.2)	
ASA 3	28 (29.5)	8 (14.8)	0.083
ITD, mm, (mean ± SD)	43.83 ± 23.33	38.30 ± 20.56	0.149
Pathologic diagnosis, *n*(%)			
PDAC	12 (12.6)	8 (14.8)	
SCN	27 (28.4)	16 (29.6)	
MCN	12 (12.6)	8 (14.8)	
SPN	25 (26.3)	11 (20.4)	
PNT	12 (12.6)	7 (13.0)	
Others	7 (7.4)	4 (7.4)	0.979
Specimen size, mm, (mean ± SD)	46.04 ± 28.15	38.81 ± 21.20	0.103
*R*0 resection, *n*(%)	94 (98.9)	54 (100.0)	1.000
Lymphatic metastasis, *n* (%)	4 (4.2)	2 (3.7)	1.000
Operative time, min, median (IQR)	210 (180–270)	240 (200–270)	0.138
Blood loss, ml, median (IQR)	100 (50–200)	100 (50–200)	0.400
FFT, days, median (IQR)	3 (3–3)	2.5 (2–3)	0.001
Diet start time, days, median (IQR)	3 (3–4)	3 (2–4)	0.002
Hospital stay, days, median (IQR)	14 (11–17)	13 (11–15)	0.051
PHS, days, median (IQR)	8 (7–11)	8 (5–9)	0.026
Reoperation, *n* (%)	2 (2.1)	2 (3.7)	0.621
Complication, *n* (%)			
Pulmonary infection	4 (4.2)	0	0.297
Abdominal infection	8 (8.4)	0	0.070
Wound infection	2 (2.1)	1 (1.9)	1.000
Pancreatic fistula	52 (54.7)	32 (59.3)	0.593
B + C fistula	24 (25.3)	15 (27.1)	0.737
Bleeding	5 (5.3)	2 (3.7)	1.000
Mortality	0	0	
CD grade 3/4, *n* (%)	8 (8.4)	3 (5.6)	0.751
Operation cost, USD, (mean ± SD)	3237.7 ± 1442.1	6998.4 ± 1314.9	<0.001
Total cost, USD, (mean ± SD)	8256.8 ± 2149.0	11522.7 ± 1569.3	<0.001

MIPD, minimally invasive distal pancreatectomy; RDP, robot-assisted distal pancreatectomy; LDP, laparoscopic distal pancreatectomy; BMI, body mass index; CA199, carbohydrate antigen 199; CEA, carcinoembryonic antigen; CA125, carbohydrate antigen 125; HB, hemoglobin; PDD, pancreatic duct dilatation; ASA, American Society of Anesthesiology; ITD, imaging tumor diameter; PDAC, pancreatic ductal adenocarcinoma; SCN, serous cystic neoplasms; MCN, mucinous cystic neoplasms; SPN, solid pseudopapillary neoplasms; PNT, pancreatic neuroendocrine tumor; FFT, first ﬂatus time; PHS, postoperative hospital stay; CD, Clavien–Dindo; USD, U.S. dollar.

**Table 2:** The preservation rate of spleen (benign and borderline neoplasms in MIPD).

	LDP (*n* = 83)	RDP (*n* = 46)	*P*
Spleen preservation, *n* (%)	42 (50.6)	36 (78.3)	0.002
Operation methods, *n* (%)			
Kimura's technique	22 (26.5)	23 (50.0)	0.007
Warshaw's technique	20 (24.1)	13 (28.3)	0.604

MIPD, minimally invasive distal pancreatectomy; RDP, robot-assisted distal pancreatectomy; LDP, laparoscopic distal pancreatectomy.

**Table 3:** The follow-up data (MIPD).

	LDP (*n* = 80)	RDP (*n* = 50)	*P*
Endocrine dysfunction, *n* (%)	15 (17.4)	9 (17.6)	0.976
Exocrine dysfunction, *n* (%)	2 (2.3)	0	0.529
Thrombocytosis	18	3	
OPSI	1	0	
Splenic infarction	0	0	
Mortality	6	1	

MIPD, minimally invasive distal pancreatectomy; RDP, robot-assisted distal pancreatectomy; LDP, laparoscopic distal pancreatectomy; OPSI, overwhelming postsplenectomy infection.

**Table 4:** Baseline characteristics, pathology data, and outcomes of patients (the first 32 versus the last 22 RDPs).

	Early experience (*n* = 32)	Late experience (*n* = 22)	*P*
Age, years, (mean ± SD)	50.72 ± 15.52	49.09 ± 13.91	0.695
Sex, *n*(%)			
Male	9 (28.1)	7 (31.8)	
Female	23 (71.9)	15 (68.2)	0.770
BMI, kg/m^2^, (mean ± SD)	24.31 ± 3.95	24.11 ± 3.08	0.845
CA199, u/ml, median (IQR)	13.9 (9.6–21.4)	10.9 (7.6–16.2)	0.311
CEA, ng/ml, median (IQR)	1.6 (1.0–2.3)	1.0 (0.5–2.5)	0.134
CA125, u/ml, median (IQR)	16.4 (12.0–22.7)	13.2 (10.3–18.2)	0.111
Albumin, g/l, median (IQR)	42.0 (40.9–44.0)	42.5 (40.4–45.8)	0.449
HB, g/l b, (mean ± SD)	128.31 ± 20.00	132.36 ± 17.48	0.445
PDD, *n*(%)	3 (9.4)	1 (4.5)	0.638
Comorbidities, *n*(%)			
Hypertension	7 (21.9)	4 (18.2)	0.741
Diabetes	2 (6.3)	2 (9.1)	1.000
ASA, *n*(%)			
ASA 1	5 (15.6)	2 (9.1)	
ASA 2	23 (71.9)	16 (72.7)	
ASA 3	4 (12.5)	4 (18.2)	0.750
ITD, mm, (mean ± SD)	37.06 ± 23.71	40.09 ± 15.19	0.600
Pathologic diagnosis, *n*(%)			
PDAC	4 (12.5)	4 (18.2)	
SCN	10 (31.3)	6 (27.3)	
MCN	6 (18.8)	2 (9.1)	
SPN	4 (12.5)	7 (31.8)	
PNT	5 (15.6)	2 (9.1)	
Other	3 (9.4)	1 (4.5)	0.548
Specimen size, mm, (mean ± SD)	38.25 ± 24.33	39.64 ± 16.11	0.816
*R*0 resection, *n* (%)	0	0	
Lymphatic metastasis, *n* (%)	0	2 (9.1)	0.161
Operative time, min, median (IQR)	240 (210–300)	200 (180–260)	0.011
Blood loss, ml, median (IQR)	100 (50–300)	90 (50–100)	0.052
FFT, days, median (IQR)	3 (2–3)	2 (2–3)	0.004
Diet start time, days, median (IQR)	3 (2–4)	3 (2–3)	0.027
Hospital stay, days, median (IQR)	13 (11–16)	11 (10–14)	0.047
PHS, days, median (IQR)	8 (5.5–9.5)	7 (5–8)	0.372
Reoperation, *n*(%)	2 (6.3)	0	0.508
Complication, *n*(%)			
Pulmonary infection	0	0	
Abdominal infection	0	0	
Wound infection	1 (3.1)	0	1.000
Pancreatic fistula	18 (56.3)	14 (63.6)	0.587
B + C fistula	7 (21.9)	8 (36.4)	0.243
Bleeding	2 (6.3)	0	0.508
Mortality	0	0	
CD grade 3 + 4, *n*(%)	3 (9.4)	0	0.262

RDP, robot-assisted distal pancreatectomy; BMI, body mass index; CA199, carbohydrate antigen 199; CEA, carcinoembryonic antigen; CA125, carbohydrate antigen 125; HB, hemoglobin; PDD, pancreatic duct dilatation; ASA, American Society of Anesthesiology; ITD, imaging tumor diameter; SCN, serous cystic neoplasms; MCN, mucinous cystic neoplasms; SPN, solid pseudopapillary neoplasms; PNT, pancreatic neuroendocrine tumor; FFT, first ﬂatus time; PHS, postoperative hospital stay; CD, Clavien–Dindo

**Table 5:** The preservation rate of spleen (the first 32 versus the last 22 RDPs) (benign and borderline neoplasms).

	Early experience (*n* = 28)	Late experience (*n* = 18)	*P*
Spleen preservation, *n* (%)	22 (78.6)	14 (77.8)	0.949
Operation methods, *n* (%)			
Kimura's technique	15 (53.6)	8 (44.4)	0.546
Warshaw's technique	7 (25.0)	6 (33.3)	0.540

RDP, robot-assisted distal pancreatectomy.

## Data Availability

Data that support the findings of this study are available on reasonable request from the corresponding author.
